This article has been retracted.

# Eupalinolide J Suppresses the Growth of Triple-Negative Breast Cancer Cells *via* Targeting STAT3 Signaling Pathway

**DOI:** 10.3389/fphar.2019.01071

**Published:** 2019-09-19

**Authors:** Chenghua Lou, Yan Chen, Jie Zhang, Bo Yang, Huajun Zhao

**Affiliations:** ^1^School of Pharmaceutical Sciences, Zhejiang Chinese Medical University, Hangzhou, China; ^2^Department of Cell and Molecular Pharmacology and Experimental Therapeutics, Medical University of South Carolina, Charleston, SC, United States

**Keywords:** eupalinolide J, triple-negative breast cancer, STAT3, apoptosis, cell cycle

## Abstract

Persistent activation of STAT3 plays an important role in the development of triple-negative breast cancer (TNBC), and suppression of STAT3 is considered as a novel approach for cancer therapy. In this project, we aimed to examine the anticancer activity and molecular mechanism of eupalinolide J (EJ) in TNBC cells. The presented results demonstrated that the growth of human TNBC cells (MDA-MB-231 and MDA-MB-468 cells) was obviously inhibited by EJ. The IC_50_ values were 3.74 ± 0.58 and 4.30 ± 0.39 μM, respectively. Further study demonstrated that EJ suppressed the proliferation of TNBC cells mainly through cell apoptosis induction, mitochondrial membrane potential (MMP) disruption, and cell cycle arrest. Meanwhile, the STAT3 and p-STAT3 in EJ-treated TNBC cells were remarkably suppressed. Importantly, silencing of STAT3 by STAT3-shRNA significantly blunted the anticancer activities of EJ in TNBC cells, suggesting that EJ suppressed cancer cell proliferation *via* targeting the STAT3 pathway. Notably, further study demonstrated that EJ significantly promoted the degradation of STAT3 in TNBC cells. Finally, EJ exhibited an effective antitumor activity against MDA-MB-231 cells *in vivo*. In conclusion, we identified that EJ suppressed the growth of TNBC cells *via* targeting the STAT3 signaling pathway. These results strongly support that EJ is a promising therapeutic agent for TNBC.

## Introduction

Breast cancer is the most common cancer in women (Siegel et al., 2018). In 2018, the number of diagnosed new cases is around 1.7 million, and the number of death is about 522,000 worldwide (Ginsburg et al., 2017). Generally, breast cancer is well-established as a heterogeneous disease in the clinic (Polyak, 2011). There are several identified types, among which the triple-negative breast cancer (TNBC) is the most fatal for patients. Conventionally, TNBC is defined by the lack of ER, PR, and HER2 in breast cancer cells (Dent et al., 2007). It is well-known for its metastatic and aggressive characteristics and poor outcome in the clinic (Wang et al., 2018a). It makes up 10∼20% of diagnosed breast cancers (Boyle, 2012). Up to now, the treatment of TNBC patients is still a challenging task due to the absence of appropriate targets for drugs.

Great effort has been made to explore novel therapies to decrease the mortality rates of patients with TNBC. The signal transducer and activator of transcription 3 (STAT3), an important transcription factor in STAT family, is demonstrated to exert an enormous function on promoting cancer proliferation, survival, metastasis, angiogenesis, and immunosuppression (Aleskandarany et al., 2016). Overexpression of STAT3 has been verified in many cancers, such as breast, lung, and liver cancers (Harada et al., 2014; Park et al., 2017; Egusquiaguirre et al., 2018). Recently, many studies had demonstrated that there were around 80% of TNBC with overexpressed STAT3 (Chun et al., 2015). Therapeutics by targeting STAT3 could potently suppress the tumor progression (Hussain et al., 2007; Lin et al., 2010). Hence, development of novel anticancer agents by targeting STAT3 could be a promising approach for the treatment of TNBC.

Natural products are a well-known treasure house for the development of novel anticancer drugs (Mann, 2002; Koehn and Carter, 2005; Newman and Cragg, 2012). *Eupatorium lindleyanum* DC., a traditional Chinese medicine, is conventionally used to treat influenza and bronchopneumonia (Yang et al., 2007). Recently, this herb has been paid more and more attention. A growing number of studies have identified antiinflammatory (Wang et al., 2018b), anticancer (Yang et al., 2016, Yang et al., 2017a; Tian et al., 2018), and antioxidant (Yan et al., 2011) activities of this herb. Eupalinolide J (EJ) (**Figure 1A**), one of the main compounds in *Eupatorium lindleyanum* DC., is demonstrated to exert inhibitory effects on STAT3 activation in our previous work (Yang et al., 2017a). However, the anticancer activity and exact molecular mechanisms of EJ against breast cancer cells are still unclear. In this project, we examined the effects of EJ on TNBC cells and elucidated its anticancer mechanism. Our results demonstrated that EJ is a promising therapeutic agent for TNBC.

**Figure 1:** EJ suppresses the growth of TNBC cells *in vitro*. **(A)** The chemical structure of eupalinolide J (EJ). **(B)** Effects of EJ on the growth of MDA-MB-231 cells. **(C)** Effects of EJ on the growth of MDA-MB-468 cells. **(D)** Effects of EJ on the growth of MCF-10A cells. Cells were incubated with EJ for 24, 48, and 72 h (24 h for MCF-10A cells). After treatment, cell viability was quantified by MTT assay. Values represent mean ± SD of three independent experiments. **P < 0.01, ***P < 0.001 vs. control group.

## Materials and Methods

### Cell Culture and Reagents

MDA-MB-231, MDA-MB-468, and MCF-10A cell lines were obtained from the Chinese Academy of Sciences. Cells were maintained in DMEM (Gibco, USA) containing 10% fetal bovine serum (FBS, Sijiqing, Hangzhou, China) at 37°C with 5% CO_2_ in an incubator.

EJ (**Figure 1A**) was isolated from *Eupatorium lindleyanum* DC. herb in our lab, as previously described (Yang et al., 2017a). The purity of EJ was above 95% (**Supplementary Figure 1**). Antibodies against STAT3 (#30835), p-STAT3 (#4113), cyclin B1 (#12231), caspase-9 (#9508), Bax (#5023), caspase-3 (#9662), c-Myc (#9402), Bcl-xl (#2764), cleaved caspase-3 (#9664), cleaved caspase-9 (#9501), Bcl-2(#2870), caspase-8 (#4790), cleaved caspase-8 (#8592), Histone H3 (#4499), and β-tubulin (#2128) were obtained from Cell Signaling Technology. Antibody against Bad (1541-1) was obtained from Abcam.

### MTT Assay

The inhibitory effects of EJ on the growth of cancer cells were evaluated by MTT assay. Cells (5 × 10^3^ cells/well) were planted into a 96-well plate for 4 h before treatment. After that, different dosages of EJ were subjected to incubate with cancer cells. After incubation, MTT reagent was added. DMSO was used to dissolve the formazan, and the absorbance was detected under a microplate reader.

### DAPI Staining

DAPI staining was performed to detect the apoptotic cell death in EJ-treated TNBC cells. Briefly, cells were planted and subsequently incubated with EJ. After incubation, cells were harvested, washed, and fixed. DAPI reagent was then applied to stain the cancer cells. Apoptosis was observed using a fluorescence microscope (Nikon, Japan).

### Annexin V-FITC/PI Double Staining Assay

Apoptotic cell death in TNBC cells was quantified by flow cytometry using an apoptosis detection kit (Becton Dickinson, USA). The assay was performed as we previously described (Lou et al., 2009).

### Evaluation of Mitochondrial Membrane Potential (MMP, Δψm)

Evaluation of MMP in cancer cells was detected using an MMP detection kit (Beyotime, China) according to the manufacturer’s instructions. The assay was performed as we previously described (Lou et al., 2009).

### Cell Cycle Assessment

The distribution of cell cycle in EJ-treated TNBC cells was examined using a propidium iodide (PI)/RNase staining kit (Becton Dickinson, USA). The assay was performed as we previously described (Tian et al., 2018).

### ShRNA Design and Transfection

ShRNAs for STAT3 were designed by Genechem (Shanghai, China). The target sequences of STAT3-shRNA were 241-ACAATCTACGAAGAATCAA-2553 and 241-CGGCAACAGATTGCCTGCATT-2553, respectively. The transfection of shRNA into breast cancer cells was performed with Lipofectamine 2000 as previously described (Xiang et al., 2017).

### Immunofluorescence Analysis

The immunofluorescence assay was performed as previously described (Kim et al., 2018).

### Nuclear Extracts Preparation

The nuclear and cytoplasmic proteins in TNBC cells were extracted using a nuclear and cytoplasmic protein extraction kit (Beyotime, Shanghai, China). The assay was performed according to the manufacturer’s instructions. Extracted fractions were collected for western blotting analysis.

### Western Blotting Analysis

Cancer cells were incubated with EJ or DMSO for 24 h. Then cells were washed and lysed in radio immunoprecipitation assay (RIPA) buffer containing phosphatase inhibitors and protease inhibitors. The total protein was extracted and quantified. Cell lysates were separated and transferred to polyvinylidene fluoride (PVDF) membrane. Then the membrane was blocked, followed by incubation with primary and secondary antibodies. After washing with PBS, enhanced chemiluminescent detection system was used for imaging detection.

### Xenograft Mouse Model

The antitumor activity of EJ *in vivo* was evaluated by a nude mouse xenograft model. BALB/c nu/nu female mice were obtained from Shanghai Experimental Animal Center (Shanghai, China). The experiment was performed as previously described in our lab (Yang et al., 2017b).

### TUNEL Staining

Fluorescent TUNEL staining (Beyotime, Shanghai, China) was performed according to the manufacturer’s instructions. The assay was performed as we previously described in our lab (Yang et al., 2017b).

### Immunohistochemistry (IHC)

IHC was used to investigate the level of STAT3 in tumor samples. The experiment was performed as we previously described (Zhu et al., 2017).

### Statistical Analysis

Results were expressed as mean ± SD of three independent experiments. Statistical differences between the groups were assessed by one-way ANOVA using SPSS 18.0 software. For the *in vivo* longitudinal tumor growth data, two-way ANOVA was used to analyze and compare the significant difference between different treatment groups. *P values < 0.05 were considered statistically significant.

## Results

### EJ Suppresses the Growth of TNBC Cells

To examine the inhibitory effects of EJ on the growth of TNBC cells, cells were incubated with various dosages of EJ for different times. Cell viability was evaluated by MTT assay. Results indicated that EJ effectively suppressed the growth of TNBC cells (**Figures 1B, C**). IC_50_ values were 3.74 ± 0.58 µM for MDA-MB-231 and 4.30 ± 0.39 µM for MDA-MB-468 at 72 h. Interestingly, compared with the TNBC cells, normal MCF-10A breast epithelial cells were less sensitive to EJ-induced cytotoxicity (**Figure 1D**).

### EJ Induces Apoptosis in TNBC Cells

As EJ showed significant inhibitory effects on the growth of TNBC cells, we next investigated whether the cell growth inhibition was a result of apoptosis induction. DAPI staining was used to detect the morphological changes in the nuclei. As shown in **Figure 2A**, after treatment with EJ or DMSO for 24 h, compared with the control groups, remarkable characteristics of apoptosis were observed in EJ-treated groups, such as nuclear fragmentation, chromatin condensation, and apoptotic bodies. In addition, EJ-induced apoptotic response in MDA-MB-231 and MDA-MB-468 cells was further confirmed by flow cytometry analysis. The number of apoptotic cells was obviously increased with EJ treatment (**Figure 2B**). These data indicated that EJ could induce apoptotic cell death in TNBC cells.

**Figure 2:** EJ induces apoptotic cell death in TNBC cells. **(A)** Effects of EJ on the nuclear morphology of TNBC cells. Fluorescence photomicrographs of TNBC cells stained with DAPI after treatment with EJ (×40). After staining, the morphology of cancer cells was observed under a fluorescence microscopy. **(B)** Flow cytometry analysis of apoptosis in TNBC cells. TNBC cells were pretreated with EJ. The number of apoptotic cells was quantified by flow cytometer. Values represent mean ± SD of three independent experiments. **P < 0.01, ***P < 0.001 vs. control group.

### EJ Disrupts MMP in TNBC Cells

As we have known, apoptosis induction through mitochondrial pathways is usually accompanied by the loss of MMP. Based on the above notion, we assessed the MMP using JC-1 fluorescence. As shown in **Figure 3**, an increase of green fluorescence could be seen in MDA-MB-231 and MDA-MB-468 cells after treatment with EJ, indicating marked reduction of MMP in cancer cells. The above data indicated that EJ induced MMP disruption in TNBC cells. As we all know, the caspases play critical roles in cell apoptosis. In the mitochondrial pathway, caspase-9 is regarded as an initiator, and caspase-3 is a critical effector in the execution of cell apoptosis. For this reason, we next examined the activation of caspase-9 and caspase-3 in EJ-treated TNBC cells. As shown in **Figure 4A**, the expression levels of cleaved caspase-3 and cleaved caspase-9 were significantly increased with EJ treatment. Furthermore, the expression levels of Bcl-2 family proteins, which control the MMP and the activation of caspase cascade, were also examined in this study. Western blotting data showed that the expression levels of Bcl-2 and Bcl-xl were visibly downregulated, whereas the expression levels of Bax and Bad were significantly upregulated (**Figure 4B**). These results implied that EJ induced TNBC cell apoptosis through the mitochondrial pathway. In addition, the activation of caspase-8 was also observed (**Figure 4A**), indicating that the extrinsic death signaling pathway was involved in EJ-induced apoptosis in TNBC cells.

**Figure 3:** EJ disrupts MMP in TNBC cells. TNBC cells were treated with EJ for 24 h. Then cancer cells were harvested and washed with ice-cold PBS. After incubation with JC-1, the MMP in TNBC cells were detected by flow cytometry. Values represent mean ± SD of three independent experiments. ***P < 0.001 vs. control group.

**Figure 4:** EJ activates intrinsic and extrinsic apoptotic pathways in TNBC cells. **(A)** Western blotting analysis of caspases in TNBC cells after treatment with EJ. **(B)** Western blotting analysis of Bcl-xl, Bcl-2, Bax, and Bad in TNBC cells after treatment with EJ. Values represent mean ± SD of three independent experiments. *P < 0.05, **P < 0.01,***P < 0.001 vs. control group.

### EJ Arrests Cell Cycle at the G2/M Phase

To determine whether EJ modulates the cell cycle among TNBC cells, the cell cycle distribution in EJ-treated cells was analyzed. As shown in **Figure 5A**, the percentage of cells at the G2/M phase was remarkably raised. Consistent with the above results, western blotting results demonstrated that the expression levels of cyclin B1and c-Mycin TNBC cells were obviously decreased, whereas the protein level of p21 was increased (**Figure 5B**). Those data indicated that EJ induced cell cycle arrest at the G2/M phase in TNBC cells.

**Figure 5:** EJ arrests cell cycle at the G2/M phase. **(A)** Cell cycle analysis by flow cytometry. Cells were pretreated with EJ. After PI staining, cell cycle distribution was analyzed. **(B)** Western blotting detection of cell cycle regulator in cancer cells. The expression levels of cyclin B1, c-Myc, and p21 in TNBC cells were analyzed by western blotting assay. Values represent mean ± SD of three independent experiments. *P < 0.05, **P < 0.01,***P < 0.001 vs. control group.

### EJ Suppresses the Growth of TNBC Cells *via* Targeting the STAT3 Pathway

As EJ was demonstrated to exert inhibitory effects on STAT3 activation in our previous study, we next determined whether EJ could suppress STAT3 in TNBC cells by western blotting assay. As shown in **Figure 6A**, the expression level of STAT3 and p-STAT3 was significantly downregulated with the treatment of EJ. To further examine whether EJ suppressed the growth of TNBC cells *via* targeting the STAT3 pathway, TNBC cells were transfected with STAT3-shRNA (shRNA-1 and shRNA-2) plasmid or negative control shRNA plasmid (NC-shRNA). As shown in **Figure 6B**, STAT3-shRNA transfection obviously decreased the expression levels of STAT3 and p-STAT3 in TNBC cells. Compared with the NC-shRNA groups, the STAT3-shRNA transfection did not significantly affect cell viability in 24 h (**Figure 6C**). Importantly, compared to the NC-shRNA groups, silencing of STAT3 by STAT3-shRNA significantly blunted the anticancer activities of EJ in TNBC cells (**Figure 6D**). These results indicated that EJ suppressed the growth of TNBC cells *via* targeting the STAT3 pathway.

**Figure 6:** EJ inhibits the growth of TNBC cells *via* targeting the STAT3 pathway. **(A)** The STAT3 expression in TNBC cells was significantly downregulated. Cancer cells were incubated with various dosages of EJ for 24 h. Then the expression of STAT3 in cancer cells was detected by western blotting assay. **(B)** Knockdown of STAT3 in TNBC cells *via* shRNA transfection. TNBC cells were transfected with STAT3-shRNAs (shRNA-1 and shRNA-2) plasmid or negative control shRNA plasmid (NC-shRNA). The expression of STAT3 in TNBC cells was determined using western blotting. **(C)** Effects of siRNAs on the cell viability of TNBC cells. The cell viability of transfected TNBC cells was determined at 24 h. **(D)** Knockdown of STAT3 in TNBC cells obviously blunted the sensitivity of TNBC cells to EJ-induced cytotoxicity. TNBC cells were transfected with (shRNA-1 and shRNA-2) or negative control (NC- shRNA) and then cultured with different concentrations of EJ. After incubation, cell viability was quantified by MTT assay. Values represent mean ± SD of three independent experiments. *P < 0.05, **P < 0.01,***P < 0.001 vs. control group.

### EJ Promotes the Degradation of STAT3 in TNBC Cells

Nuclear translocation of STAT3 is essential for its function as a transcription factor (Liu et al., 2005). Therefore, the immunofluorescence assay was performed to investigate the nuclear translocation of STAT3. However, our results demonstrated that EJ significantly promoted the degradation of STAT3 in cytoplasm instead of blocking the nuclear translocation (**Figure 7A**). Meanwhile, the nuclear and cytoplasmic fractions of protein lysate from the EJ-treated cells were separated. Upon the EJ treatment, the protein levels of STAT3 and p-STAT3 in nuclei and cytoplasm were significantly decreased in TNBC cells (**Figure 7B**). These results indicated that EJ promoted the degradation of STAT3 in TNBC cells.

**Figure 7:** EJ promotes the degradation of STAT3 in TNBC cells. **(A)** Immunofluorescence analysis of STAT3 in EJ-treated TNBC cells. The localization of STAT3 (red) and DAPI (blue) in TNBC cells. Cancer cells were treated with EJ (15 µM) for 24 h. STAT3 was probed with primary antibody and labeled using secondary antibody conjugated. **(B)** STAT3 expression in the nucleus or cytoplasm was detected using western blotting. Cells were treated with different concentrations of EJ for 24 h. Then the nuclear and cytosol fractions of protein lysate from treated cells were separated. Histone H3 was used as a nuclear loading control. β-tubulin was used as a cytoplasmic loading control. Values represent mean ± SD of three independent experiments. *P < 0.05,**P < 0.01, ***P < 0.001 vs. control group.

### EJ Suppresses Tumor Growth in a Nude Mouse Xenograft Model

To further assess the effects of EJ on tumor growth *in vivo*, a nude mouse xenograft model transplanted with MDA-MB-231 cells was used in this study. As shown in **Figures 8A–D**, compared with the vehicle groups, EJ significantly suppressed tumor growth *in vivo*. Notably, there was no significant difference in body weight in all groups, indicating that the compound did not have obvious toxicity *in vivo* (**Figure 8C**). Moreover, compared to the vehicle groups, TUNEL staining results showed that EJ significantly increased the number of TUNEL-positive cells, indicating apoptotic cell death in tumors (**Figure 8E**). Furthermore, the IHC analysis demonstrated that EJ significantly reduced the expression level of STAT3 in the tumor tissue sections (**Figure 8E**). The above data implied that EJ could effectively suppress the growth of tumor *in vivo*.

**Figure 8:** EJ inhibits tumor growth in mouse xenograft models. **(A)** Tumor imaging. BALB/c nude mice were inoculated with MDA-MB-231 cells and treated with EJ (20 mg/kg, intraperitoneally) for 20 days. After sacrifice, the tumor imaging was recorded. **(B)** The tumor volume was measured during the experiment. **(C)** The change of body weight was recorded. **(D)** The tumor weight was recorded after sacrifice. **(E)** TUNEL staining and IHC analysis of tumor sections in control and EJ-treated groups. TUNEL staining results showed that EJ significantly increased the number of TUNEL-positive cells, indicating apoptotic cell death in tumors. IHC analysis demonstrated the low expression of STAT3 in groups with EJ treatment. Values represent mean ± SD of three independent experiments. *P < 0.05,**P < 0.01, ***P < 0.001 vs. control group.

## Discussion

Therapeutic options to breast cancer vary depending on the different subtypes (Parise and Caggiano, 2014). Generally, recommended treatments for luminal A and luminal B breast cancers include chemotherapeutic agents, anti-HER2 treatments, and endocrine therapy (Parise and Caggiano, 2014), and for HER2^+^ breast cancers, anti-HER2 agents in combination with other cytotoxic chemotherapy are the conventional options (Burnett et al., 2017; Ponde et al., 2018). However, there were limited treatment options for TNBC patients, as they do not benefit from the traditional therapies.

Recently, the targeted therapies have been widely recommended to treat TNBC patients. However, still only a few patients benefit from those therapies. The investigation of effective targets for TNBC therapy is still a challenging work. A potential candidate biomarker is STAT3, which has been strongly implicated in cancer cell proliferation, angiogenesis, and metastasis (Bromberg and Darnell, 2000; Bromberg, 2002). In the current study, we demonstrated that EJ showed significant inhibitory effects on the growth of TNBC cells both *in vitro* (**Figure 1**) and *in vivo* (**Figure 8**). Suppression of STAT3 was remarkably observed in EJ-treated TNBC cells and tumor samples (**Figures 6A** and **8E**). Importantly, knockdown of STAT3 in TNBC cells obviously blunted the sensitivity of TNBC cells to EJ-induced cytotoxicity (**Figures 6B, D**), which suggested that STAT3 was directly involved in EJ-induced cell death. Moreover, promoted degradation of STAT3 in cancer cells by EJ was verified (**Figure 7**).

Apoptosis induction is one of the main manners by which many anticancer agents suppress cancer cell growth. There are two pathways: the extrinsic and intrinsic pathways. In the intrinsic pathway, the Bcl-2 family proteins, such as proapoptotic proteins (Bad and Bax) and antiapoptotic proteins (Bcl-2 and Bcl-xl), play important roles in apoptosis induction (Duan et al., 2019). In response to proapoptotic signals, BH3-only and Bcl-2 family proteins will be activated, followed by an efflux of cytochrome c and activation of caspases (McArthur and Kile, 2018). Finally, the apoptosis process takes place. According to the reports, Bcl-2 and Bcl-xl have been verified as direct targets of STAT3 (Siddiquee et al., 2007). Constitutively active STAT3 upregulates the survival factors, Bcl-2, Bcl-xl, and Mcl-1 (Catlett-Falcone et al., 1999; Epling-Burnette et al., 2001; Bhattacharya et al., 2005). Disruption of STAT3 signaling pathways leads to the inhibition of Bcl-xl, Mcl-1, and Bcl-2 (Catlett-Falcone et al., 1999; Epling-Burnette et al., 2001; Bhattacharya et al., 2005) and activates the expression of the proapoptotic protein Bax (Nielsen et al., 1999) in cancer cells. Consistent with the above notion, in the present study, accompanied by the suppression of STAT3, EJ treatment resulted in a significant induction of apoptosis in TNBC cells (**Figures 2** and **8E**). Meanwhile, disruption of MMP (**Figure 3**), activation of cleaved caspase-3 and -9 (**Figure 4A**), downregulation of Bcl-2 and Bcl-xl (**Figure 4B**), and upregulation of Bax and Bad (**Figure 4B**) were obviously observed in EJ-treated TNBC cells. These data demonstrated that EJ induced the apoptosis of TNBC cells *via* the intrinsic pathway. In addition, in the extrinsic pathway, Fas and TRAIL are the most intensively studied members of the death receptor family. Fas and TRAIL receptors can promote caspase activation by recruiting caspase-8 (Wilson et al., 2009). It has been demonstrated that STAT3 and c-Jun can bind the Fas gene (TNFRSF6) in a complex to repress Fas expression (Ivanov et al., 2001). Interestingly, the activation of caspase-8 was demonstrated by western blotting in this study (**Figure 4A**), suggesting that the extrinsic pathway was also involved in EJ-induced apoptosis. The activation of the extrinsic pathway in TNBC cells could contribute to the suppression of STAT3 by EJ.

Numerous studies have verified that STAT3 exerted an enormous function on cell proliferation induced by cytokines (Bromberg and Darnell, 2000; Bromberg, 2002; Yu et al., 2009). Especially the cell cycle regulators (cyclin D1 and cyclin B), which participate in cell cycle regulation, are directly regulated by STAT3 (Sinibaldi et al., 2000; Jarnicki et al., 2010). Persistent STAT3 activation resulted in inducing overexpression of target genes, such as cyclin D1 and cyclin B1 (Yang et al., 2005). Inhibition of STAT3 in cancer cell lines was correlated with downregulation of cyclin B1, cyclin D1, and c-Myc (Bollrath et al., 2009; Zhao et al., 2011). In the present project, we verified that the cell cycle in EJ-treated TNBC cells was arrested at the G2/M phase (**Figure 5A**). The expression levels of cyclin B1 and c-Myc in TNBC cells were obviously downregulated (**Figure 5B**), which are key cell cycle regulators at the G2/M phase. Meanwhile, p21, a potent cyclin-dependent kinase inhibitor and a target gene of STAT3 (Siveen et al., 2014), which can induce cell cycle arrest at the G2/M phase *via* suppressing cyclin B/cdc2, was significantly upregulated (**Figure 5B**). These results demonstrated that induction of cell cycle arrest could be another mechanism of EJ against TNBC cells.

Finally, the antitumor activity of EJ *in vivo* was verified in a nude mouse xenograft model transplanted with MDA-MB-231 cells. EJ significantly suppressed the tumor growth *in vivo* without obvious toxicity (**Figures 8A–D**). Meanwhile, the reduction of STAT3 in EJ-treated groups was also observed (**Figure 8E**). However, further work is still needed, including evaluation of the anticancer activity of EJ in other TNBC cell lines both *in vitro* and *in vivo* model systems.

## Conclusions

In conclusion, this study has documented the anticancer activity of EJ on TNBC cells. Our results demonstrated that EJ suppressed the growth of TNBC cells *via* targeting the STAT3 signaling pathway. EJ suppressed the growth of TNBC cells mainly through apoptosis induction, cell cycle arrest, and MMP disruption. The results of this study indicate that EJ is an effective anticancer agent for TNBC therapy in the future.

## Data Availability

All datasets generated for this study are included in the manuscript and/or **Supplementary files**.

## Ethics Statement

The animal studies were approved by the Institutional Animal Care and Use Committee (IACUC) of Zhejiang Chinese Medical University (No ZSLL-2013-108). All applicable international, national, and/or institutional guidelines for the care and use of animals were followed. All procedures performed in studies involving animals were in accordance with the ethical standards of the institution or practice at which the studies were conducted.

## Author Contributions

CL, BY, and HZ designed the study. CL, YC, and BY performed the experiments. CL, YC, and JZ analyzed the data and wrote the manuscript. All authors read and approved the final manuscript.

## Funding

This research was funded by the Zhejiang Provincial Natural Science Foundation of China (no. LY17H310007 and Y17H280004 and LZ15H310001), Natural Science Foundation of China (no. 81774003 and 81773868), the first level (HZ) in Zhejiang Province “151 talents project” and Qianjiang Scholar Program funded by Zhejiang Province (HZ).

## Conflict of Interest Statement

The authors declare that the research was conducted in the absence of any commercial or financial relationships that could be construed as a potential conflict of interest.

## Abbreviations

EJ, eupalinolide J; DMSO, dimethyl sulfoxide; MTT, 3-(4,5-dimethyl-2-thiazolyl)-2,5-diphenyl-2H-tetrazolium bromide; STAT3, signal transducer and activator of transcription 3; NF-κB, nuclear factor-κB; FBS, fetal bovine serum; DMEM, Dulbecco’s modified Eagle’s medium; PVDF, polyvinylidene fluoride; IHC, immunohistochemistry; PBS, phosphate buffered saline; MMP, mitochondrial membrane potential; TNBC, triple-negative breast cancer; MAPK, mitogen-activated protein kinase; ER, estrogen receptor; PR, progesterone receptor; HER2, human epidermal growth factor receptor 2; DAPI, 4’,6-diamidino-2-phenylindole; PI, propidium iodide; NC, negative control.
